RETRACTED

# Eleutheroside E alleviates cerebral ischemia-reperfusion injury in a 5-hydroxytryptamine receptor 2C (Htr2c)-dependent manner in rats

**DOI:** 10.1080/21655979.2022.2071009

**Published:** 2022-05-03

**Authors:** Zheng Liu, Wenwei Gao, Yuanqin Xu

**Affiliations:** Department Of Neurology, The Second Affiliated Hospital of Baotou Medical College, Inner Mongolia University of Science & Technology, Baotou, Inner Mongolia, China

**Keywords:** Ischemia-reperfusion, eleutheroside E, htr2c, rat hippocampal neuron, apoptosis

## Abstract

Stroke is the central disorder underlined by ischemia-reperfusion (I/R) injury. Eleutheroside E (EE) is administered as the shield in some ischemia tissues with anti-inflammatory action. However, whether EE defends I/R-induced damage in the brain remains unknown. Here, we demonstrated that EE significantly alleviated the cerebral I/R injury and reduced the apoptosis of hippocampal neuron cells in rats. During the anti-apoptosis process, EE significantly upregulated the expression of 5-hydroxytryptamine receptor 2C (Htr2c) gene. Silencing Htr2c expression dramatically weakened the protective effect of EE on I/R-induced apoptosis of rat hippocampal neuron. EE-regulated Htr2c also remarkably inhibited the expression of caspase-3, −6 and −7, thereby suggesting a plausible anti-apoptosis mechanism associated with Htr2c/caspase axis. These findings elicit the potentially clinical strategy that targets Htr2c to improve outcome of ischemia brain.

## Highlights

- Eleutheroside E relieved the cerebral I/R injury 35.
- Eleutheroside E protected hippocampal neuron cells against apoptosis.
- Eleutheroside E up-regulated the Htr2c expression.
- Eleutheroside E inhibited caspase activities through Htr2c.

## Introduction

Ischemia-Reperfusion (I/R) injury is stated as the dramatically damaged by the reperfusion of proximal blood into tissues with ischemia or oxygen depletion and thereby causes multiple organ dysfunctions, including stroke and arrhythmias [1]. I/R-derived stroke is the ruling cause of disability and the NO. 2 cause of death worldwide [2].The first recognition of I/R injury was recorded at 1972 in studying the coronary artery [3]. Since that, scientists have been attempting to dissect the cause of I/R injury. Blood resupply into brain with ischemic condition initially changes several cellular metabolism and resultantly triggers inflammatory response, oxidative stress, and apoptosis basically through the excess of mitochondrial reactive oxygen species (ROS), and following activation of innate immunity partially mediated by PPAR-γ [4], while it is also essential for survival [5]. At the cellular level, activating toll-like receptor 4 signaling pathway contributes to global cerebral I/R-induced neuronal death in the hippocampal formation [6]. Recently, many studies revealed that microRNAs are critical regulators of neuronal survival during cerebral I/R injury [7,8]. Although these biological responses to reperfusion are established, the detailed molecular mechanisms of I/R injury in the brain are not well understood, therefore impeding effective therapy.

RETRACTED

Increasing studies have demonstrated that natural compounds from herbal have potent protection against I/R injury [9–11]. Fucoidan, a sulfated polysaccharide based predominantly on L-fucose, ameliorates hepatic I/R injury in mice via JAK2/STAT1-mediated apoptosis and autophagy [12]. Also, a natural product isolated from *Curcuma longa*, Curcumin, limits oxidative stress, inflammation, mitochondria dysfunction, liver Kupffer cells (KCs) activation to reduce I/R injury [13,14]. Eleutheroside E (EE) is one major bioactive component of *Eleutherococcus senticosus* (ES), a known tonic and sedative herb that has multiple health benefits according to anciently medical record [15]. EE administration enhances endurance performance and improves physical fatigue, strong protection against nerve cell death and neuritic atrophy, and dramatic function of anti-inflammation by suppressing the action of pro-inflammatory mediators [16–19]. However, little is known about the effect of this compound and correlated cellular mechanism on the improvement of I/R-induced injury in the brain.

Amongst all the brain regions (including the cerebrum, cerebellum, hypothalamus, and hippocampus) studied, the pyramidal neurons of the hippocampus are perceptively assailable to ischemic injuries [20–22] and die during the first days of reperfusion [23–25], which may eventually result in the retrograde amnesia [26]. However, whether EE mediates the I/R-induced apoptosis in rat hippocampal neuron cells is unknown.

Given all above mention, we hypothesized that EE might have protective role on I/R-injured brain and anti-apoptosis activity on hippocampal neuron cells induced by I/R injury. To address these questions, we chose the cerebral I/R model in rats. We firstly investigate the overall protection of EE in rat brain and rat hippocampal neuron cells injured by I/R. Further, we mechanistically explored that EE inhibits the I/R-induced apoptosis of rat hippocampal neuron cells and ultimately relieve cerebral I/R injury through upregulating Htr2c expression.

## Materials and methods

### Generation of cerebral I/R model in Rats

For cerebral I/R induction, the previously described protocol that occluded middle cerebral artery (MCA) utilizing a modification of the intraluminal technique was introduced into adult male Sprague-Dawley rats (body weight 180–210 g) [2,27]. In brief, a total of 42 rats were randomly assigned into I/R and sham groups. The MCA of rats (*n* = 14 per group) were performed by bilateral clamping to generate ischemia. 2 h post ischemia, bilateral clamping was gently removed to achieve the resupply of cerebral blood flow. In sham-operated animals (*n* = 14), the utilization of the clamps was omitted and all other procedure was performed. The animal work was carried out by fully following to the regulations in the Guide for the Care and Use of Laboratory Animals of the National Institutes of Health. Animal Research Ethics Committee of Baotou medical college approved the current animal protocol [Approval No. SYXK(MENG)2018–0003]. One day after operation, the rats were scored for neurological deficits according to the Longa 5-point Scale [28]. Briefly, this neurological examinations were performed daily until sacrifice. A score of 0 indicated no neurologic deficit, a score of 1 (failure to extend left forepaw fully) indicated a mild focal neurologic deficit, a score of 2 (circling to the left) indicated a moderate focal neurologic deficit, and a score of 3 (falling to the left) a severe focal deficit; rats with a score of 4 did not walk spontaneously and had a depressed level of consciousness. Rats with score of 1–3 were selected for further experiments while dead rats or those with scores of zero or 4 were excluded, and random backup rats were chosen to fill in the slots. Specifically, first 7 rats in each group were applied in 2,3,5-Triphenyltetrazolium chloride (TTC) staining. Parts of brain tissues of another 7 rats were used for H&E and TUNEL staining, while the rest of tissues were stored at −80°C for western blotting, quantitative RT-PCR assay, and other measurements.

RETRACTED

### Eleutheroside E (EE) treatment

A purity of ≥ 98% (HPLC) of EE (CAS: 39,432–56-9) was commercially available by Sigma Aldrich. 1% sodium carboxymethylcellulose (CMC-Na) was used to dissolve the EE at 1 mg/ml before utilization [29]. For treatment, both the EE (10 mg/kg) and vehicle were fed once a day by gavage from day 1 to day 21 after the induction of cerebral I/R. Two days post the last administration of EE or vehicle control, rats were anesthetized and the brain was isolated. The hippocampi was separated from brain for both application of H&E staining and single cell isolation, and coronary brain sections were sliced from the brain for histological analysis.

### Histological analysis

To carefully dissect the cerebral infarct of the affected brain tissue, a commonly available method, TTC staining was carried out to identify the infarction volume on 2 mm thickness of coronal brain sections [2]. In brief, the I/R-injured or sham-operated brains were immediately removed from rats and then coronal sections were performed at 2 mm intervals from the rostrum to caudal. All slices were soaked in a 1% TTC buffer at 37°C. After 20 min incubation, a computerized image analysis system (Biovis Image Plus) was employed to scan and analyze coronal brain sections stained by TTC. The infarct area of all brain sections of I/R-injured or sham-operated rats were analyzed and multiplied by section thickness to obtain the infarct volume.

4% neutral paraformaldehyde (Sigma-Aldrich) was used to fix the sliced brain tissues. The fixed tissues were then embedded in paraffin, sectioned, and finally stained with hematoxylin and eosin for examining the pattern, shape, and structure of cells after I/R injury. At least 40 consecutive fields under microscopy with ×400 magnification were used to quantify the histopathological score.

### Apoptosis detection by flow cytometry

The hippocampi were obtained as previously described with a slight modification [30–33]. The dissected hippocampi were transferred into 15 ml Falcon tubes with papain buffer (0.1 mg/ml papain, 2 μg/ml DNase, 200 μg/ml DL-Cysteine HCl, 200 μg/ml BSA, and 5 mg/ml glucose) for 10 min at 37°C. After discarding the papain buffer by pipetting, tissues were triturated by a fire-polished glass pipette for 10 time in a trituration medium (1 μg/ml DNase in HBSS buffer). The supernatant was collected and transferred into new 15 ml Falcon tubes without disturbing the un-dissociated tissues. The trituration were repeated for three times and the pooled supernatant was centrifuged for 5 min at 150 g, 4 ^o^C. For staining, a single-cell suspension of hippocampal neuron cells isolated from rats administrated by I/R or I/R plus EE was prepared in harvested buffer (0.05% trypsin, 0.02% EDTA, 0.05% glucose) [34]. After digesting, a small amount of cells were plated in 12-well plates pretreated with 0.1% poly-D-lysine. With indirect anti-NeuN immunocytochemistry assay, each well in 12-well plates demonstrated 99% neuronal cells [35]. Also, the digested cells were operated by continuously washing in PBS twice and eventually re-suspending in binding buffer containing 10 mM HEPES, 140 mM NaCl, 2.5 mM CaCl2 at pH 7.4. A final concentration of 200 ng/ml of Annexin V-FITC was loaded to suspended cells. 10 min post incubation in the dark at room temperature, samples were washed in PBS and re-suspended in 190 µl of binding buffer. Prior to flow cytometric analysis, 10 µl of PI was added to each sample. Stained cells were subjected into FACStar plus flow cytometer (Becton Dickinson). The ratio of fluorescence intensities excited at 488 nm was detected at an emission wavelength of 560 nm for PI and 515 nm for FITC. Cell Quest software (Becton Dickinson) was utilized to analyze the data analysis.

RETRACTED

### CCK-8 assay

Cell viability was analyzed by using CCK-8 assay kit (Dojindo) according to manufacturer introductions. In particular, isolated hippocampal neuron cells were incubated in the medium containing 10 µl CCK-8 reagent at 37°C for 1 h. The viable cell numbers were evaluated by measurement of absorbance at 450 nm.

### Gene chip probe array analysis

Total RNA isolation from hippocampal neuron cells of I/R and I/R plus EE samples was performed by utilizing Trizol (Gibco BRL). RNA cleanup by RNeasy Kit (Qiagen) was detected by the Agilent 2100 Bioanalyzer. The concentration of RNA was determined by spectrophotometer at 260 nm absorbance. The first-strand cDNA synthesis was reverse-transcribed using a T7 promoter-containing oligo(dT) primer. Following RNase H-mediated second-strand cDNA synthesis, the double-stranded cDNA was purified and serves as a template in the resultant in vitro transcription (IVT) reaction. The IVT reaction is carried out in the presence of T7 RNA polymerase and a biotinylated nucleotide analog/ribonucleotide mix for complementary RNA (cRNA) amplification and biotin labeling. After cleanup and quantification of biotin-labeled cRNA, the metal-induced hydrolysis was introduced to fragment those cRNA into 35 to 200 base fragments. To screen the genes, the samples were hybridized to the Rat Genome arrays (U230A) for 16 h at 45°C to Gene Chip test analysis [36]. Then we washed, stained the arrays with streptavidin-phycoerythrin, and scanned with the Gene Array scanner (Affymetrix). Affymetrix Microarray Suite 5.0 (MAS) software was used to analyze the data.

### RNA interference

The synthesis of small interference RNA (siRNA) for Htr2c was customized by Qiagen. Three Htr2c siRNAs (100 nM for each) were transfected into hippocampal neuron cells by using Lipofectamine 3000 (Invitrogen) [37], respectively. A negative control, scrambled siRNA (siRNA-NC) was also transfected into same cells to investigate the effect of Htr2c on the I/R-injured brains by subsequently quantitative RT-PCR and western blotting assay.

### Quantitative RT-PCR Assay

Total RNA isolated by above-mentioned protocol was applied for quantitative RT-PCR assay. The first-strand cDNA generated by was generated by a commercially available kits (Applied BioSystems) using 2 μg of total RNA. Then 7 Universal PCR Master Mix (Applied Biosystems) was applied to all subsequent PCR reaction. All transcriptional expression levels were standardized against GAPDH. Primer pairs used in this study were as follows: GAPDH: 5’-CCTTCATTGACCTCAACTAC-3’ and 5’-GGAAGGCCATGCCAGTGAGC-3’ [38]; Htr2c: 5’-T ATCGCTGGACCGGTATGTAGC-3’ and 5’-GCAATCTTCATGATGGCCTTAGTC −3’; caspase-3: 5’-GGTATTGAGACAGACAGTGG-3’ and 5’-CATGGGATCTGTTT CTTTGC-3’; caspase-6: 5’-TTCAGACGTTGACTGGCTTG-3’ and 5’-TCCAG CTTGTCTGTCTGGTG-3’; caspase-7: 5’-TTTGCTTACTCCACGGTTCC-3’ and 5’- GAGCATGGACACCATACACG-3’. All amplifications were at least 3 technically and 3 biologically replicated.

RETRACTED

### Western blotting analysis

For immunodetection of Htr2c and caspase 3, 6, and 7, the lysate of hippocampal neuron cells were obtained by directly incubating cells in the protein buffer (50 mM pH 7.5 Tris-HCl, 0.5% SDS, 150 mM NaCl, 1% sodium deoxycholate, and 1 mM PMSF) for 30 min [39,40]. All proteins supernatant were clarified by centrifugation (13,000 × g, 30 min, 4°C). After protein concentration quantification, 50 µg of total proteins was separated on a 12% SDS-PAGE and then transferred onto nitrocellulose membranes in a transfer instrument containing transfer buffer (25 mM Tris-HCl, 195 mM glycine, and 20% (v/v) methanol). Ponceau S staining evaluated the transfer efficiency of proteins. Membrane blocking was fulfilled by 3% (w/v) bovine serum albumin (BSA) dissolved in buffer containing pH 8.0 50 mM Tris, 150 mM NaCl, and 0.05% Tween 20 for 1 h at room temperature. All primary antibodies used in current study were a rabbit polyclonal anti-caspase 3 (A0214, ABclonal, 1:2000), a rabbit polyclonal anti-caspase 6 (A1784, ABclonal, 1:2000), and a rabbit polyclonal anti-caspase 7 (A1524, ABclonal, 1:2000). The secondary antibody was a goat anti-rabbit IgG (AS070, ABclonal, 1:15,000). The intensities of positive protein band were collected and analyzed by Fujifilm LAS-3000 imager.

### ROS production, malondialdehyde (MDA), superoxide dismutase (SOD) and glutathione (GSH) peroxidase measurements

Intracellular ROS production measured as previously described [41]. Briefly, treated cells were further incubated with 10 μM DCFH-DA at 37°C in a CO_2_ incubator for 20 minutes. Cells were then washed three times with 200 μL of DMEM to get rid of any residual DCFH-DA, after which 100 μL of DMEM was added to each well. The fluorescent intensity was immediately determined spectrophotometrically using a SpectraMax M5 (Molecular Devices, CA, USA) with an excitation wavelength of 488 nm and an emission wavelength of 525 nm. The level of emitted fluorescence was correlated with the quantity of ROS in the cells. Each measurement was performed in duplicate, and cellular fluorescence intensities were expressed as fold changes relative to the Control group. The MDA content and the SOD and GSH peroxidase activity levels in cultured cells were determined using commercially available MDA, SOD, and GSH peroxidase kits following the manufacturer’s instructions. The data were analyzed spectrophotometrically using a SpectraMax M5 (Molecular Devices, CA, USA).

RETRACTED

### Statistical analysis

All data were expressed as means ± SEM and subjected to be performed the statistical analysis using GraphPad Prism 7.04 (GraphPad Software, Inc., USA). The one-way ANOVA with Turkey’s multiple comparison test was used to analyze statistical significance among groups. Significant differences were calculated by indicated statistical methods. The *P-*value with two significant levels (0.05 and 0.01) was presented [42].

## Results

This study used the cerebral I/R model in rats to explore the protective role of Eleutheroside E (EE) in brain I/R damage. We hypothesized that EE could protect the nervous system function and ameliorate I/R injury. Further molecular regulation mechanism of EE and its modulation of biomarker genes and signal pathways were also determined.

### Eleutheroside E (EE) attenuates I/R-induced apoptosis in rat hippocampal neuron

We firstly explored the effect of EE administration on the I/R-induced infarct in rat brain sections. Interestingly, TTC staining suggested that EE significantly reduced 15% volumes of I/R-induced infarction (Figure 1 a and b). Figure 1c shows representative histological micrographs of brains from each group. Sections from the sham-operated (Control) rat brain presented the normal histology and cerebral cell vacuolization, the swelling and necrosis extensively occurred in I/R rats. These changes were obviously reversed when EE was given before I/R (Figure 1c). Typically, apoptosis of hippocampal neuron cells accounts for the serious extent of I/R injury in the brain [22,26]. So we next investigate whether EE mediates the I/R-induced apoptosis of hippocampal neuron cells. Figure 1d shows representative histological micrographs of hippocampus from each group. In contrast to the sham-operated group, hippocampal neurons from I/R group displayed as severe damage, with nuclear deformation, cellular swelling, and scattered arrangement, as well as characteristic changes of apoptosis. The administration of EE dramatically reversed above-mentioned damages, demonstrating by the complete and tightly arranged hippocampal neurons, clear nucleoli with a uniform staining, and the transparent cytoplasm (Figure 1d). Using the enhancement of Annexin V-FITC intensity as an indicator for convincing apoptosis (Gating strategy was shown in Supplementary Fig. 1), we discovered that hippocampal neuron cells treated with EE had a markedly lower cell apoptosis than cells injured by I/R (Figure 1e and 1f). The CCK-8 assay showed that cell viability was significantly increased in I/R+ EE group compared to I/R group (Figure 1g). These data suggest that EE can alleviate the cerebral I/R injury by reducing the apoptosis of hippocampal neuron cells.

RETRACTED

**Figure 1.** **The protective effect of EE on cerebral I/R injury and apoptosis of hippocampal neuron cells**. (a) Effect of EE on infarct volume of rat brain subjected to I/R injury. (b) Infarction ratios from **(A)** were presented as mean ± SEM. (c) Light microscopy photomicrographs depicting sections from brain of rats receiving sham operation, I/R, or I/R plus EE. (d) Light microscopy photomicrographs depicting sections from hippocampus of rats receiving sham operation, I/R, or I/R plus EE. (e) Apoptosis analysis of hippocampal neuron cells in rats treated with sham operation, I/R, or I/R plus EE. (f) The apoptosis rate from **(E)**. (g) CCK-8 assay of hippocampal neuron cells in rats treated with sham operation, I/R, or I/R plus EE. Error bars ± SEM, *p < 0.05.

### EE suppresses the expressions of caspase 3, 6, and 7 in hippocampal neuron cells

TUNEL staining revealed the obvious apoptosis in I/R-injured coronary brain tissue and hippocampus section compared to the control section, and EE administration could ameliorate this I/R-induced apoptosis in both coronary brain and hippocampus tissues (Figure 2 a and b). Since cell apoptosis was commonly triggered by the activation of caspase cascades [43,44] and EE refrains the I/R-induced apoptosis, the activity of caspase 3, caspase 6, and caspase 7 were therefore assessed by RT-PCR and western blotting. Initially, I/R induced the upregulated expression of caspase 3, 6, and 7 in transcriptional and protein levels (Figure 2 c and d). After the administration of EE into I/R rats, these caspase proteins were all restored to the normal level (Figure 2 d and e).

**Figure 2.** **The apoptosis in I/R-injured brain and hippocampus tissues and the expressions of caspase 3, 6, and 7 in I/R-treated hippocampal neuron cells could be relieved by EE administration**. (a) Representative images of TUNEL staining for coronary brain tissues receiving sham operation, I/R, or I/R plus EE. (b) Representative images of TUNEL staining for hippocampus tissue receiving sham operation, I/R, or I/R plus EE. The expression analysis of caspase 3, 6, and 7 both in mRNA (c) and protein (d) levels in hippocampal neuron cells of I/R-treated rats in the absence and presence of EE by real time PCR and western blotting. (e) The relative density of protein level of caspase 3, 6, and 7 from **(D)**. Data were presented as mean ± SEM, **p < 0.01.

RETRACTED

### EE functions as an anti-oxidant in hippocampal neuron cells

As shown in Figure 3a to 3d, i/R injury significantly increased the ROS and MDA levels and decreased SOD and GSH activities in primary hippocampal neuron cells isolated from rats, suggesting the induction of oxidative stress by I/R in such cells. Interestingly, I/R-injured rats administered with EE has almost similar level of all these indicators to control rats in hippocampal neuron cells, demonstrating that EE has an anti-oxidative function.

**Figure 3.** **EE has an anti-oxidative effect on I/R-treated hippocampal neuron cells**. EE administration reduced the ROS production (a) and MDA content (b) and increased the activities of SOD (c) and GSH peroxidase (d) on I/R-induced hippocampal neuron cells. Data were presented as mean ± SEM, **p < 0.01.

### EE inhibits Htr2c expression in hippocampal neuron cells

To further identify the anti-apoptosis molecular mechanism, we use the gene array to screen the downstream signaling molecules of EE. Thirty-eight genes that have relatively crucial relation with hippocampal neuron cells by searching literature [45–47] were selected to analysis, and ultimately, as expected, a majority of these genes expression had been changed in cells in response to EE treatment (Figure 4a). In principle, for the above genes, abundance was dramatically upregulated in the cells that benefit for anti-apoptosis (or vice versa). Thus, we primarily focus on the genes which can be enhanced by EE treatment. One of the seven upregulated proteins, Htr2c, had the highest expression, indicating that Htr2c may be a central downstream target of EE. Then we confirmed the Htr2c expression in EE-treated cells from mRNA and protein levels. In transcriptional level, untreated cells expressed a basic level of Htr2c, while the expression of Htr2c markedly induced in hippocampal neuron cells of rats treated with EE (Figure 4b). This finding suggested that EE can boost Htr2c expression. We also examine the protein level of Htr2c. As shown in Figure 4c and 4d, EE could really enhance the Htr2c production in treated cells compared to the untreated cells.

**Figure 4.** **EE-treated hippocampal neuron cells show enhanced expression of Htr2c**. (a) Unsupervised hierarchical clustering of thirty-eight vital genes in hippocampal neuron cells of I/R-treated rats in the absence and presence of EE. (b) The mRNA expression of Htr2c in the presence of EE. (c) The protein expression of Htr2c in the presence of EE. (d) The relative density of protein level of Htr2c from **(C)**. Data were presented as mean ± SEM, **p < 0.01.

### Htr2c is responsible for the anti-apoptosis action of EE

To examine the mechanism that links Htr2c to the anti-apoptosis activity of EE, RNA interference was employed to downregulate the production level of Htr2c. Three synthetic siRNA that target Htr2c were applied, and relative expression of Htr2c was measured in transcriptional and translational levels. Transcriptional level assay demonstrated that siRNA worked for Htr2c as its level was markedly suppressed, and siRNA-Htr2c-3 represented the best inhibitory effect (Figure 5a). In line with the transcriptional assay, the downregulation pattern of Htr2c expression in protein level was occurred by Htr2c siRNAs (Figure 5b and 5c), especially for siRNA-Htr2c-3. Because the administration of EE boosted the expression of Htr2c, the knock-downed effect of Htr2c on EE-treated hippocampal neuron cells was analyzed. Similar to the above outcome, hippocampal neuron cells of rats treated by I/R plus EE had lower apoptosis in contrast to that in I/R. However, EE-treated cells inhibiting Htr2c expression prevented the decreased apoptosis resulted from siRNA-Htr2c-3 treatment (Figure 5d and 5e), thereby indicating the specificity of anti-apoptotic function of Htr2c. These observations suggest that Htr2c seems to be a crucial downstream signal effector for EE in treatment with I/R-induced apoptosis of rat hippocampal neuron.

RETRACTED

**Figure 5.** **Htr2c contributes to anti-apoptosis effect of EE on I/R-treated hippocampal neuron cells**. (a and b) The expression analysis of Htr2c both in mRNA (a) and protein (b) levels in hippocampal neuron cells treated with siRNA-Htr2c-1 to 3 by real time PCR and western blotting. (c) The relative density of protein level of Htr2c from **(B)**. (d) The apoptosis analysis of hippocampal neuron cells of I/R rats treated simultaneously without or with EE and EE plus siRNA-Htr2c-3. (e) The apoptosis rate from **(D)**. Data were presented as mean ± SEM.

### Htr2c is a potential target for EE to suppresses the expression of caspase 3, 6, and 7

To examine a becoming possibility that Htr2c regulates the caspase 3, 6, and 7 expressions in EE-administered hippocampal neuron cells upon I/R, we use siRNA-Htr2c-3 to knocked down the expression level of Htr2c. Interestingly, in the mRNA level, the expression of caspase 3, 6, and 7 was detected to be higher in EE plus siRNA-Htr2c-3-administered cells as compared to cells expressed scrambled siRNA or not (Figure 6a). More critical, caspase expression of EE plus siRNA-Htr2c-3-administered cells was similar almost with that in hippocampal neuron cells of I/R rats. Also, we discovered a similar pattern of caspase 3, 6, and 7 expressions in protein level (Figure 6b). The protein level of Bax (pro-apoptotic) was increased and Bcl2 (anti-apoptotic) was reduced by I/R injury, which were reversed by EE treatment (Figure 6b and 6c). Again, Htr2c siRNA blocked the effect of EE by increasing Bax expression and decreasing Bcl2 expression in EE-treated cells (Figure 6b and 6c). These data suggest that Htr2c is a potentially downstream target for EE to mediate the expression of caspase proteins.

RETRACTED

**Figure 6.** **EE inhibits the expressions of caspase 3, 6, and 7 through Htr2c**. (a) The expression analysis of caspase-3, −6 and −7 in mRNA levels in hippocampal neuron cells of I/R rats treated simultaneously without or with EE, EE plus siRNA-NC, and EE plus siRNA-Htr2c-3. (b) Western blotting of caspase-3, −6 and −7, Bax, and Bcl2 in hippocampal neuron cells of I/R rats treated simultaneously without or with EE, EE plus siRNA-NC, and EE plus siRNA-Htr2c-3. (c) The relative density of protein level of caspase 3, caspase 6, caspase 7, Bax, and Bcl-2 from **(B)**.Data were presented as mean ± SEM, *p < 0.05, **p < 0.01.

## Discussion

Numerous attempts in prevention largely decrease stroke incidence and mortality [48,49]; however, less strategies have been developed to decline the detrimental outcomes of cerebral ischemia. Transient global cerebral ischemia results in cell apoptosis or death of hippocampal neurons after reperfusion, which in turn, exacerbates brain injury [23,25,50]. Although it has been reported that *E. senticosus*, a main herb for the isolation of EE, may develop a neuroprotective effect against ischemic injury in brains [51], whether the mechanism underlying this neuroprotection has a relationship with apoptosis is sealed. The outcomes of the present study demonstrate the crucial role of EE in the survival of neurons after I/R injury. In follow-up experiments, we also introduce the mechanistic link between EE and its anti-apoptosis function.

The central finding in our study is that EE suppresses the apoptosis of hippocampal neuron cells upon I/R. Apoptosis is an active form of cell death, which is intimately bound up with differentiation of gene expression [52]. Currently, we show that EE regulates the Htr2c expression, and Htr2c involved in anti-apoptosis action of EE through inhibiting the expression of caspase 3, 6, and 7, thereby demonstrating a plausible anti-apoptosis mechanism associated with Htr2c/caspase axis.

Htr2c is a major one relevant and identified receptor for recognizing 5-hydroxytryptamine, also known as serotonin, in both human and animal studies [53]. Previous studies have demonstrated the close relationship between mental illnesses and serotonin deficiencies [54], and also found that Htr2c is a neuromodulator that involves in psychiatric behaviors such as clinical depression [55,56]. Depression is the most resultant and harmful affective disorder following stroke [57]. Genetic analysis reveals that Htr2c polymorphism appears to be involved in the pathogenesis of post-stroke depression [58], providing an imaginable clue to study the function of Htr2c in I/R-induced brain neuron injury. Our present study finds that Htr2c contributes to the anti-apoptosis action of EE in hippocampal neuron cells. This is a novel finding because previous studies did not ferret out any inter-relationship among EE, Htr2c, and apoptosis.

RETRACTED

Htr2c gene encodes a cell multi-pass membrane protein that binds to multiple PDZ domain proteins, which is widely produced in the brain, to provoke its clustering [59,60]. Furthermore, after extracellular ligand binding, it can trigger signaling via association with nucleotide-binding proteins (G proteins) that activate the down-stream effectors, including phosphatidylinositol-calcium second messenger system [53]. The latter improves the export of Ca^2+^ ions from intracellular stores and modulates the activity of phosphatidylinositol 3-kinase and downstream signaling events [61,62]. In the current, the down-stream targets of anti-apoptosis of EE-mediated Htr2c in hippocampal neuron cells are three members of the caspase family, caspase 3, 6, and 7. Although apoptosis regulated by caspase 3, 6, and 7 has been extensively documented in the literature [63–65], the ability of Htr2c to reverse cell death through the regulation of caspase proteins is previously unrecognized.

## Conclusion

We have broadly deciphered that EE modulates the I/R-induced apoptosis of hippocampal neuron cells through influencing caspase 3, 6, and 7 expressions by upregulation of Htr2c expression. This event is the potential cause of alleviative I/R injury in rat brain upon EE administration. More importantly, our study provides new and valuable cognition toward the development of a complete understanding of the pathogenesis of I/R-induced brain injury. This elicits the potential that Htr2c may be a thinkable clinical target for those I/R-mediated stroke patients in the future.

## Supplementary Material

Supplemental Material

## Data Availability

Data available on request.
